# Chest Computed Tomography Images in Neonatal Bronchial Pneumonia under the Adaptive Statistical Iterative Reconstruction Algorithm

**DOI:** 10.1155/2021/6183946

**Published:** 2021-10-27

**Authors:** Ying Sun, Liao Wu, Zhaofang Tian, Tianping Bao

**Affiliations:** ^1^Department of Neonatology, The Affiliated Huai'an No. 1 People's Hospital of Nanjing Medical University, Huai'an 223300, Jiangsu, China; ^2^Department of Neurology, The Affiliated Huai'an No. 1 People's Hospital of Nanjing Medical University, Huai'an 223300, Jiangsu, China

## Abstract

This study was to explore the application value of chest computed tomography (CT) images processed by artificial intelligence (AI) algorithms in the diagnosis of neonatal bronchial pneumonia (NBP). The AI adaptive statistical iterative reconstruction (ASiR) algorithm was adopted to reconstruct the chest CT image to compare and analyze the effect of the reconstruction of CT image under the ASiR algorithm under different preweight and postweight values based on the objective measurement and subjective evaluation. 85 neonates with pneumonia treated in hospital from September 1, 2015, to July 1, 2020, were selected as the research objects to analyze their CT imaging characteristics. Subsequently, the peripheral blood of healthy neonates during the same period was collected, and the levels of C-reactive protein (CRP) and erythrocyte sedimentation rate (ESR) were detected. The efficiency of CT examination, CRP, ESR, and combined examination in the diagnosis of NBP was analyzed. The results showed that the subjective quality score, lung window subjective score, and mediastinal window subjective score were the highest after CT image reconstruction when the preweight value of the ASiR algorithm was 50%. After treatment, 79 NBP cases (92.9%) showed ground-glass features in CT images. Compared with the healthy neonates, the levels of CRP and ESR in the peripheral blood of neonates with bronchial pneumonia were much lower (*P* < 0.05). The accuracy rates of CT examination, CRP examination, ESR examination, CRP + ESR examination, and CRP + ESR + CT examination for the diagnosis of NBP were 80.7%, 75.3%, 75.1%, 80.3%, and 98.6%, respectively. CT technology based on AI algorithm showed high clinical application value in the feature analysis of NBP.

## 1. Introduction

Neonatal bronchial pneumonia (NBP) is the most common pediatric pneumonia disease caused by mycoplasma infection, accounting for about 10% of neonatal pneumonia. Because of the anatomical and physiological characteristics of the neonatal respiratory tract and the immune characteristics of the body, the morbidity and mortality of bronchial pneumonia in children are significantly increased compared with adults, and its clinical symptoms are different. It is still one of the important diseases threatening the health of newborns [1]. According to the statistics of the causes of neonatal death of the World Health Organization (WHO) from 2000 to 2003, bronchopneumonia accounted for 19%, which is the first cause of neonatal death; the incidence of NBP in developed countries is 0.05 times/person/year. In developing countries, the incidence of NBP is 6 times that of developed countries, and the anatomical characteristics of children and the sensitivity of individuals to drugs are different. Approximately 2.4 million children die every year. NBP caused by multiple pathogens and physical and chemical factors is still threatening the health and life of newborns [2]. At present, pneumonia still ranks first in the neonatal prevalence and mortality in our country. Therefore, it is necessary to explore the diagnosis and treatment methods of NBP, further improve the diagnosis and treatment of NBP, promote the early recovery of children, and reduce the pain of children. Most of the NBP treated with regular drugs have good results, but some children with pneumonia only rely on conventional drugs to treat the results poorly. Therefore, the diagnosis and treatment of neonatal pneumonia still need to be further explored [3]. There are many diagnostic methods for NBP, such as fiberoptic bronchoscopy and bronchography. CT imaging has also been used in the diagnosis of NBP and has a certain diagnostic value [4] with the rapid development of imaging technology. However, CT scan is highly radioactive. In order to reduce its impact on neonates' health, low-dose CT is often used clinically to diagnose pediatric diseases. Low-dose CT scanning reduces the radiation while increasing the noise in the image, which affects the diagnosis accuracy of the disease to a certain extent [5, 6].

The ASiR (an AI algorithm) has been introduced in recent years to balance the quality of CT image and radiation dose, and it has been proven to significantly improve the image quality and reduce the radiation dose of CT scans [7–9]. Compared with the filtered back projection (FBP) algorithm, the ASiR algorithm can reconstruct high-quality CT images with low noise and less artifacts [10], because the traditional iterative reconstruction algorithm runs slowly and the modified ASiR algorithm can effectively weight FBP data and ASiR data to fuse, while reducing the image noise and increasing the processing speed [11].

Based on this, the AI ASiR algorithm was introduced firstly in this study to reconstruct the low-dose chest CT images of neonates, and then the CT characteristics and clinical features of neonates with bronchial pneumonia were analyzed. In addition, the accuracy of different methods for the diagnosis of bronchial pneumonia was analyzed and compared. This study was intended to provide a reference for improving the clinical diagnosis rate of NBP.

## 2. Basic Theories of CT Reconstruction

### 2.1. Physical Basis of CT Reconstruction

The CT imaging process mainly used different energy waves as radiation sources to perform projection of the object after irradiation, so as to obtain the reconstructed object [12]. The radiation source of CT imaging was mostly X-ray or *γ*-ray. X-ray was selected as an example to explain the principle of CT image reconstruction. When X-rays passed through an object, they would gradually attenuate in the body of the object. The density of the constructed object was different, so the attenuation speed of X-ray was also different. For objects with a more homogeneous medium, the attenuation of X-rays obeyed the Lambert–Beer theorem [13]:

(1) $$\begin{array}{c} I=I_{0}e^{-\mu x}, \end{array}$$

where *I* refers to the intensity after the attenuation of the ray through the object, *I*_0_ represents the intensity when the ray was incident, *μ* is the attenuation coefficient, and *x* refers to the transmission length.

For inhomogeneous object, the attenuation coefficient *μ* could be regarded as a function of *x* and *y*; that is, *μ* = *μ* (*x*, *y*). Therefore, the total attenuation of the ray that can pass through the object along path *L* in a certain direction *i* could be expressed as follows:

(2) $$\begin{array}{c} \int_{L}\mu \;di=\ln\left(\frac{I_{0}}{I}\right). \end{array}$$

### 2.2. Mathematical Basis of CT Reconstruction

The mathematical basis of CT image reconstruction was the Radon transformation (as shown in Figure 1) and the inverse transform theory proposed by the Austrian Mathematician Radon in 1917 [14].

As given in Figure 1, the calculation equation of straight line *L* in the plane *xoy* could be written as follows:

(3) $$\begin{array}{c} L:s=x\;\cos\;\varphi +y\;\sin\;\varphi , \end{array}$$

where *s* represents the distance from origin *O* to straight line *L*, and *φ* represents the angle between the normal of straight line *L* and the *x*-axis (positive direction).

The mathematical expression of the line integral value of the attenuation function *f* (*x*, *y*) along straight line *L* could be written as follows:

(4) $$\begin{array}{c} R_{f}\left(s,\varphi \right)=\int_{L}f\left(x,y\right)\text{d}l, \end{array}$$

where *R* refers to the Radon transformation of the attenuation function, which could be expressed as *R*_*f*_.

The coordinate system *xoy* was rotated counterclockwise by *φ* degrees along origin *O* to obtain a new coordinate system *x*′*oy*′. Then, the parameter equations of *x* and *y* of straight line *L* in this coordinate system are given as follows:

(5) $$\begin{array}{c} \left\{\begin{array}{c} x=x^{\prime }\;\cos\;\varphi -y^{\prime }\;\sin\;\varphi ,\\ y=x^{\prime }sin\varphi +y^{\prime }cos\varphi . \end{array}\right) \end{array}$$

After equation (5) was incorporated into equation (4), the Radon transformation of the attenuation function could be performed in a rotating coordinate system, which could be written as follows:

(6) $$\begin{array}{c} R_{f}\left(s,\varphi \right)=\int_{-\infty }^{\infty }\left(x^{\prime }\;\cos\;\varphi -y^{\prime }\;\sin\;\varphi ,x^{\prime }\;\sin\;\varphi +y^{\prime }\;\cos\;\varphi \right)dy^{\prime }. \end{array}$$

The process of Radon inverse transformation was the process of CT image reconstruction, which required to calculate the target object density based on projection data. The specific calculation equation of Radon inverse transformation is shown as follows:

(7) $$\begin{array}{c} f\left(r,\theta \right)=\frac{1}{2\pi^{2}}\int_{0}^{\pi }\int_{-\infty }^{\infty }\frac{1}{r\;\cos\left(\theta -\varphi \right)-s}\frac{\partial R_{f}\left(s,\varphi \right)}{\partial s}\text{d}s\text{d}\varphi . \end{array}$$

where *f* (*r*, *θ*) is the polar coordinate representation of the attenuation function.

Equation (7) was conversed to obtain the convolution form. The polar coordinate representation of the converted attenuation function could be written as *f*(*r*, *θ*)=(1/2*π*)∫_0_^*π*^*dφ*  (*R*_*f*_′(*s*, *φ*)*∗*(1/*πx*_*r*_))_*x*_*r*_=*r*cos(*θ* − *φ*)_, where *∗* is convolution and (1/*πx*_*r*_) refers to the convolution factor of Hilbert transform.

## 3. Methods

In this study, 85 NBP patients treated in our hospital from September 1, 2015, to July 1, 2020, were selected as the research objects. Firstly, all children underwent a CT imaging examination. After the examination, the CT images were processed using AI algorithms, and the quality of the processed CT images would be independently evaluated by two radiologists with at least 5 years of work experience. After that, 85 newborn children with pneumonia and 95 healthy children were checked for biochemical indicators, and the biochemical indicators of the two groups of children were compared. Finally, all research data were collected, and the biochemical indicators of the two groups of children were statistically analyzed. The sensitivity, specificity, and accuracy of CT diagnosis were analyzed and compared. The detailed research methods were as follows.

### 3.1. Research Objects

85 cases of pneumonia neonates treated in hospital from September 1, 2015, to July 1, 2020, were selected as the research objects: 48 males and 37 females. 95 healthy children who underwent physical examination at the hospital during the same period served as the control group. The families of all had been clarified about the radioactivity of CT examination and the risks of enhanced examinations before the examination and had signed the informed consent forms. All examinations in this trial had been approved by the Medical Ethics Committee of the hospital.

### 3.2. Imaging Examination

The scan range of the image was strictly set. Brilliance 64-slice spiral CT (128 slices) was used to scan from the top to the bottom of the child's chest to the diaphragmatic level of the lung base. After the consent of neonates' family members, CT scan was performed in neonates' quiet state to remove the metal material on the chest to avoid the appearance of image artifacts. 0.5 mmBp lead clothing was adopted to cover the lower abdomen and pelvic cavity of the neonate, and the neonate was required to keep a supine position for chest CT scan. During the scanning, the specific parameters of the CT scan were set according to the requirements for chest low-dose scan of neonates. The tube voltage was 100∼120 kV, the tube current was 50 mA, the speed was 0.8 s/rot, the pitch was 1.375 : 1.000, the noise index was 12, the layer thickness was 5 mm, and the spacing was 5 mm.

### 3.3. CT Images Process Based on AI Algorithm

The CT images obtained from low-dose scans were reconstructed using the AI ASiR and FBP algorithms. The preweight value of ASiR was set to 0%, 10%, 20%, 30%, 40%, 50%, 60%, 70%, 80%, 90%, and 100% to evaluate the reconstructed image with the ASiR algorithms. The preweight value was turned off to optimize the subjective scores of the mediastinal window and lung window so that they both could reach the highest preweight values, based on which the postweight value interval of the ASiR algorithm was set in turn. The percentage indicated the proportion of iterative reconstruction. When the proportion was 0%, it meant that the FBP algorithm was used for image reconstruction, and when the proportion was 100%, it meant that the ASiR algorithm was used for image reconstruction. The type of image reconstruction had to select a standard algorithm, and the reconstructed layer thickness was set to 1.25 mm.

### 3.4. Quality Evaluation of Reconstructed CT Image

The chest CT image was uploaded to the workstation for observation. The region of interest (ROI) was selected in the lung field, aorta, paraspinal soft tissue, and vertebral body in the upper (sternoclavicular joint layer), middle (pulmonary vein layer), and lower (near diaphragmatic muscle layer) parts of the axial CT image, and the ROI = 100 mm^2^. The CT values (represented by ROIa and ROIm) and the density standard deviations (SD) of different ROI regions were recorded, and the average of the CT values of the 3 slices was calculated and adopted. The noise and contrast-to-noise ratio (CNR) in the reconstructed image were detected and calculated, respectively, of which CNR could be calculated with CNR = (ROIa/ROIm)/SD. When it was required to extract ROI regions in images of different levels, it was necessary to ensure that the position, size, and shape of the ROI were consistent.

2 radiologists with at least 5 years of work experience were selected for independent subjective evaluation of CT images. The mediastinal window and lung window were observed and scored. The scoring criteria were defined as follows. If the image reconstruction quality was very poor so that it could not be used for the clinical diagnosis of the disease, 1 point was scored; 2 points meant that the image reconstruction quality was relatively poor and could not meet the basic requirements of clinical disease diagnosis; 3 points indicated that image reconstruction quality was relatively average and basically could meet the requirements of clinical disease diagnosis; 4 points indicated that the image reconstruction quality was good and could meet the clinical requirements for the diagnosis requirements of the above diseases; and 5 points were awarded for the good image reconstruction quality, which could fully meet the diagnosis requirements of the clinical diseases. When the total score of the image evaluation exceeded 3 points, the image could be used in the clinical diagnosis of the disease. If there were any different opinions between the 2 radiologists, this could be solved by negotiation.

### 3.5. Biochemical Indicators Examinations of Neonates

The venous blood had to be collected from all neonates. The neonate was required to fast with water 10 hours before blood collection. After 10 mL of venous blood was collected, the ESR level was detected according to Widman's method, and the CRP level was detected using an automatic biochemical analyzer. The normal level of ESR was 0∼10 mm/h, and the normal level of CRP was >10 mg/L.

### 3.6. Statistical Analysis

The SPSS 22.0 statistical software package was adopted to process and analyze the test result data. The Kappa test was used to detect the consistency of the subjective scoring results of CT images. Kappa ≤0.4 was regarded as poor consistency, Kappa = 0.4–0.75 was regarded as good consistency, and Kappa ≥0.75 was regarded as excellent consistency. The single-factor ANOVA was applied to compare the image score results after reconstruction with different weights of the ASiR algorithm, and the LSD method was selected for pairwise comparison. The differences in the basic data and biochemical indicators of the two groups of neonates were compared using the independent-samples *t*-test, and the differences in the basic data and diagnosis accuracy of CT, biochemical indicators, and CT combined biochemical indicators of the two groups of neonates were compared using the chi-square test. When *P* < 0.05, the difference was statistically significant.

## 4. Results

### 4.1. Impacts of Preweight Value on Reconstructed Image Quality Based on ASiR Algorithm

The image noise and CNR changes after reconstruction of chest CT images using different preweight values (0%, 10%, 20%, 30%, 40%, 50%, 60%, 70%, 80%, 90%, and 100%) of ASiR algorithm were analyzed firstly (as shown in Figure 2). With the gradual increase of the preweight value, the noise value in the CT image showed a gradually decreasing trend, while the CNR value showed a gradually increasing trend.

Secondly, the differences between the subjective noise and subjective quality score of the image were compared after the chest CT image was reconstructed with the ASiR algorithm with different preweight values (0%, 10%, 20%, 30%, 40%, 50%, 60%, 70%, 80%, 90%, and 100%), and the results are illustrated in Figure 3. With the gradual increase of the preweight value of the ASiR algorithm, the subjective noise score in the reconstructed CT image showed a gradual decline, indicating that the noise in the reconstructed CT image was gradually reduced during the operation of the ASiR algorithm. With the gradual increase of the preweight value of the ASiR algorithm, the subjective quality score of the reconstructed CT image did not show a gradual upward trend. When the preweight value was 0%∼50%, the subjective quality score increased gradually; the subjective quality score showed a gradual decline trend when the preweight value was 50%∼100%. Among them, the subjective quality score of the CT image was the highest after reconstruction with the ASiR algorithm with 50% preweight value.

Then, the difference between the mediastinal window subjective score and lung window subjective score was compared when the chest CT image was reconstructed using the ASiR algorithm with different preweight values (0%, 10%, 20%, 30%, 40%, 50%, 60%, 70%, 80%, 90%, and 100%), and the analysis results are revealed in Figures 4 and 5, respectively. The changes in the mediastinal window and lung window subjective scores of the CT images after reconstruction were basically the same as the changes in the subjective quality score. When the preweight value was 40%∼60%, the mediastinal window and lung window subjective scores of the CT images reconstructed by the ASiR algorithm were obviously higher. Among them, the mediastinal window and lung window subjective scores of the CT image after reconstruction by the ASiR algorithm with a preweight value of 50% were the highest.

### 4.2. Impacts of Postweight Value on Reconstructed Image Quality Based on ASiR Algorithm

The above results revealed that the reconstructed CT image quality was the best when the preweight value in the ASiR algorithm was 50%. Therefore, the preweight value in the ASiR algorithm was set to 0% and 50% to compare and analyze the impacts of different postweight values on the CT value of different positions after CT image reconstruction. As shown in Figure 6, the CT value of lung tissue after reconstruction using the ASiR algorithm under different preweight values showed a gradual downward trend with the increase of postweight value. The CT value of lung tissue under 50% of preweight value was obviously lower than that under the 0% of the preweight value when the postweight value was 50%∼100%, as illustrated in Figure 6(a). With the increase of postweight value, the CT value of the vertebral body and aorta after reconstruction of the ASiR algorithm under different preweight values showed a gradual decrease, but the CT value of paraspine soft tissue was not changed greatly. The CT values of the vertebral body, aorta, and paraspine soft tissue under the preweight value of 50% were all less than those under the preweight value of 0% (as shown in Figures 6(b)–6(d)).

The impacts of ASiR algorithm on the SD value of the target position after reconstruction of the CT image under different postweight values were analyzed and compared, and the results are given in Figure 7. With the increase of postweight value, the SD value of lung tissue after reconstruction with ASiR algorithm at 0% preweight value was not obvious, while that after reconstruction with ASiR algorithm at 50% preweight value showed a trend of first increasing and then decreasing. Among them, the SD value of lung tissue under 70% postweight value was the largest (as disclosed in Figure 7(a)). As the postweight value increased, the SD values of the vertebral body, aorta, and paraspine soft tissue in CT images after reconstruction with different preweight values of the ASiR algorithm showed gradual declines. The SD values of the vertebral body, aorta, and paraspine soft tissue after reconstruction with the ASiR algorithm under 0% preweight value were much lower than those under the 50% preweight value (as shown in Figures 7(b)–7(d)).

### 4.3. CT Characteristics of NBP

The CT images of 2 neonates were undertaken as examples to analyze the characteristics of CT images (Figure 8). In the CT image of neonate A, a large area of increased density shadow could be clearly observed in the lower right lobe of the lung, the internal density was not uniform, and the air shadow of the bronchus could be clearly observed. In the CT image of neonate B, patchy and ground-glass shadows could be clearly observed in the left lower lobe of the lung, and the characteristics of bronchial inflation could be seen.

The characteristics of CT images of 85 neonates with bronchial pneumonia were analyzed (as shown in Table 1). The ground-glass CT imaging characteristic accounted for the highest proportion, followed by nodular/small air cavity consolidation, and the vascular bundle thickening also accounted for more than 50%.

### 4.4. Characteristics of Biochemical Indicators of NBP

The differences between the levels of CRP and ESR in peripheral blood of healthy neonates and neonates with bronchial pneumonia were compared, and the results are illustrated in Figure 9. The levels of CRP and ESR in peripheral blood of neonates with bronchial pneumonia were 27.3 ± 3.5 mg/L and 19.1 ± 3.7 mm/h, respectively. The levels of CRP and ESR in peripheral blood of healthy neonates were 2.7 ± 2.4 mg/L and 6.1 ± 4.8 mm/h, respectively. After comparison, it was found that the CRP and ESR levels in peripheral blood of neonates with bronchial pneumonia were remarkably lower in contrast to the healthy neonates (*P* < 0.05).

### 4.5. Analysis of the CT Value and Biochemical Indicators in the Diagnosis of Bronchial Pneumonia

The specificity, sensitivity, and accuracy of CT examination, CRP examination, ESR examination, CRP + ESR examination, and CRP + ESR + CT examination in the diagnosis of NBP were analyzed and compared. As suggested in Figure 10, the accuracies of CT examination, CRP examination, ESR examination, CRP + ESR examination, and CRP + ESR + CT examination to diagnose the NBP were 80.7%, 75.3%, 75.1%, 80.3%, and 98.6%, respectively.

## 5. Discussion

Bronchial pneumonia is the most common infectious disease in infants and young children, caused by bacteria, viral infection, or colds [15]. Due to the gradual deepening of air pollution, there are more and more pathogenic bacteria that cause diseases, and the resistance of infants and young children is lower, so the younger neonates are more susceptible to bronchial pneumonia. The main clinical manifestations of the disease are mostly fever, chills, cough, headache and general malaise, fatigue, loss of appetite, nausea, vomiting, and diarrhea. The symptoms are not serious, but they are more common. However, as the symptoms worsen, there will be symptoms such as coughing, and, in infants and young children, there are symptoms such as wheezing or difficulty breathing. In severe cases, there will be extrapulmonary manifestations, such as the nervous system, digestive system, blood system, muscles, and bones. Such abnormalities are more common in mycoplasma pneumonia. The pathogenesis of *mycoplasma pneumonia* is not very clear, mainly including respiratory epithelial adsorption, direct invasion of *Mycoplasma pneumoniae*, and the theory of immunological disorders [16, 17].

At present, imaging methods such as X-ray, chest CT, and bronchography are clinically used in the diagnosis of bronchial pneumonia [18]. As a kind of invasive examination, bronchography is of little value in newborn children. Therefore, X-ray and chest CT are often used in newborns. In previous studies of *Mycoplasma pneumoniae* lung X-ray results, only the consolidation of lung lobes/pulmonary segments and diffusely infiltrated mesh nodules can be clearly distinguished. The current study found that the results of pathological slices showed changes in bronchial inflammation and lobular consolidation, and chest X-rays could not show corresponding image changes. In the lung CT scan, the changes in bronchial inflammation such as the central nodules of the lobules can be clearly distinguished, and the patchy shadows and the pneumonia images with ground-glass changes can also be seen. Based on the lung CT thin-slice plain scan, it was known that more than two images presented in the above X-rays. At the same time, the “tree bud sign” and “tree fog sign” formed by the point and sheet infiltration formed in the early stage of the disease and the “double track sign” formed by the thickening and inflation of the bronchial wall formed by airway mucosal damage can also be affected. It can be clearly observed that uniform ground-glass changes can be clearly distributed in lung CT images. In summary, chest CT is the best examination method among neonatal pneumonia bronchial examinations. However, CT scan has high radiation. In order to reduce its impact on children's health, low-dose CT is often used clinically to diagnose pediatric diseases. Low-dose CT scanning reduces the radiation but at the same time increases the noise in the image, which affects the diagnosis accuracy of the disease to a certain extent. With the continuous update and iteration of computer network technology, various image processing technologies have also been rapidly developed and penetrated into all walks of life. Various AI algorithms have also been applied and developed in the field of medical imaging. The iterative reconstruction algorithm under AI can achieve noise control through the description and expression of noise characteristics, so it has been widely used in the reconstruction of low-dose CT imaging, of which the ASiR algorithm is the most widely used [19–22]. Therefore, the effect of CT image reconstruction using the ASiR algorithm under AI was evaluated through subjective evaluation and objective measurement firstly. The results showed that, compared with the FBP algorithm, the noise of the CT image after reconstruction by the ASiR algorithm was dramatically reduced and the quality score was improved greatly. When the preweight value was 50%, the reconstruction of the CT image by the ASiR algorithm showed the best effect. When the preconditions of the ASiR algorithm are determined, the postweight value can affect the objective indicators of the image and the supervisor's score. It was found in this study that, with the increase of postweight value, the SD values of the vertebral body, aorta, and paraspine soft tissue decreased obviously, while the SD value of lung tissue did not change much. This may be due to the heterogeneity of the lung tissue itself.

Subsequently, the CT characteristics of neonates with bronchial pneumonia were analyzed, and the results showed that ground-glass features accounted for the largest proportion, followed by nodular/small patchy air cavity consolidation and vascular bundle thickening. Ground-glass can show increased lung density and blurred edges; part of it shows the distribution of full title pages; and the pathological basis is the appearance of a small amount of serous and inflammatory exudate in the alveoli [23]. The nodular/small patchy air cavity consolidation mainly shows small patches of increased density, occupying almost all acinars and lobules [24]. In addition, the changes in serum CRP and ESR levels of neonates were detected in this study. Serum CRP is a systemic inflammatory response protein, which can reflect the infection status of neonates [25]. ESR is a nonspecific marker for the evaluation of tissue inflammation and destruction, which can reflect the aggregation state of the fibrinogen and immunoglobulin of patients [26]. The results of this study revealed that neonates with bronchial pneumonia showed greatly increased CRP and ESR levels, indicating that they suffered from systemic inflammatory response. In addition, the diagnostic accuracy on neonates with bronchial pneumonia using only CRP or ESR levels was only about 75%, while that of CRP + ESR + CT examination could be as high as 98.6%.

## 6. Conclusion

In this study, the CT images of NBP patients were reconstructed based on the AI ASiR algorithm, and it was applied in combination with the detection of serum CRP and ESR levels in the diagnosis of NBP. It was found in this study that the AI ASiR algorithm can significantly improve the quality of CT images of NBP, and CT technology based on the AI ASiR algorithm can be used in the clinical diagnosis of bronchial pneumonia in children, but the efficiency of identifying bacterial and viral pneumonia was still low and had to be improved. The diagnostic method combining CT scan and serum CRP and ESR level detection had significantly improved the sensitivity, specificity, and accuracy of disease diagnosis. This study provided reference and basis for the early diagnosis and treatment of NBP in children. However, there were still some shortcomings in this study. For example, it only analyzed the influence of the preweight and postweight values on the reconstruction effect of the AI ASiR algorithm, and the influence of other parameters on the image quality needed to be considered in the follow-up. In addition, it only analyzed the CT characteristics of NBP in children. In the follow-up, the sample size needed to be further expanded to explore the differences and diagnostic efficiency in CT characteristics of bacterial and viral NBP.

## Figures and Tables

**Figure 1:** Radon transformation.

**Figure 2:** Objective evaluation results of CT images after reconstruction using the ASiR algorithm with different preweight values. (a) Noise (HU); (b) CNR.

**Figure 3:** Comparison of subjective noise and quality score of CT images reconstructed by ASiR algorithm with different preweight values. (a) Subjective noise score; (b) subjective quality score.

**Figure 4:** Comparison of the mediastinal window subjective scores of CT images after reconstruction of the ASiR algorithm with different preweight values. (a) CT image; (b) subjective lung window score.

**Figure 5:** Comparison of subjective mediastinal window scores of CT images reconstructed by ASiR algorithm with different preweight values. (a) CT image; (b) subjective mediastinal window score.

**Figure 6:** Changes in CT values of various tissues after reconstruction of the ASiR algorithm under different postweight values.

**Figure 7:** Changes in SD values of each tissue after reconstruction of the ASiR algorithm under different postweight values.

**Figure 8:** CT images of 2 neonates with NBP.

**Figure 9:** Comparison of (a) CRP and (b) ESR levels in peripheral blood between the two groups of neonates.

**Figure 10:** Comparison of the efficiency of different methods for diagnosing NBP.

**Table 1:** The characteristic distribution of CT images of neonates with bronchial pneumonia.

CT characteristics	Cases (*n* = 85)	Percentage
Ground-glass	79	92.9
Nodular/small air cavity consolidation	74	87.1
Vascular bundle thickening	56	65.9
Atelectasis	34	40.0
Pleural effusion	27	31.8
Swollen lymph nodes	22	25.9
Large sheet consolidation	21	24.7

## Data Availability

The data used to support the findings of this study are available from the corresponding author upon request.
